# A Method for Expanding the Training Set of White Blood Cell Images

This article has been retracted.

**DOI:** 10.1155/2022/1267080

**Published:** 2022-11-09

**Authors:** Yang Su, Yu Zang, Qichen Su, Ling Peng

**Affiliations:** ^1^School of Computer and Information, Dongguan City College, Dongguan 523419, China; ^2^Department of Hematology, Huizhou First Hospital, Huizhou 516000, China; ^3^School of Mathematics and Statistics, Huizhou University, Huizhou 516000, China

## Abstract

In medicine, the count of different types of white blood cells can be used as the basis for diagnosing certain diseases or evaluating the treatment effects of diseases. The recognition and counting of white blood cells have important clinical significance. But the effect of recognition based on machine learning is affected by the size of the training set. At present, researchers mainly rely on image rotation and cropping to expand the dataset. These methods either add features to the white blood cell image or require manual intervention and are inefficient. In this paper, a method for expanding the training set of white blood cell images is proposed. After rotating the image at any angle, Canny is used to extract the edge of the black area caused by the rotation and then fill the black area to achieve the purpose of expanding the training set. The experimental results show that after using the method proposed in this paper to expand the training set to train the three models of ResNet, MobileNet, and ShuffleNet, and comparing the original dataset and the method trained by the simple rotated image expanded dataset, the recognition accuracy of the three models is obviously improved without manual intervention.

## 1. Introduction

Human blood contains components such as plasma, red blood cells, white blood cells, and platelets. Although white blood cells only account for 0.2% of whole blood, they play an important role in protecting human health [1]. White blood cells are generally divided into neutrophils, eosinophils, basophils, monocytes, and lymphocytes [2], and changes in these cell counts can be used as the basis for diagnosing certain diseases or evaluating the therapeutic effect of certain diseases [3–9]. Therefore, the accuracy and efficiency of white blood cell detection and classification are very important for the auxiliary diagnosis of diseases [10].

The traditional method of white blood cell classification is mainly the staining method, which stains blood cells and then identifies and counts them under a light microscope [11]. This method has a large workload, low efficiency, and high requirements for practitioners, and the effect of classification and counting is easily affected by human factors [12]. At present, there are many computer-aided methods for the classification and counting of white blood cells. Early computer-aided methods were mainly based on morphology, in which the shape, color, and other characteristics of white blood cells are artificially analyzed, and morphological processing is used to separate white blood cells from the background to achieve the purpose of classification, such as the method proposed in the literature [13–16]. With the development of machine learning technology, some machine learning-based white blood cell classification methods have emerged.

The main work of these methods is to design a model, use the training set to train it, get a model that performs better on the training set, and then use the test set to test the classification effect of the model. For example, Patil et al. used the CCA (canonical correlation analysis) method based on the CNN-LSTM network structure to address the issues of multiple cells overlap to improve the recognition accuracy [17]; Su et al. used morphological correlation operations to extract the characteristics of white blood cells and then brought them into three kinds of neural networks to achieve the purpose of classification [18]; Jiang et al. proposed a new CNN model combining a batch normalization algorithm and residual convolution structure [19]; Liang et al. proposed a CNN-RNN framework to fully extract image features recursively to achieve better classification accuracy [20]. When there is enough computation and dataset, machine learning can replace the manual extraction of image features and can have higher efficiency than complex programming to extract image features manually [21].

The classification effect of machine learning is affected by the number of samples in the training set. When the number of samples in the training set is small, the problem of underfitting will occur [22], resulting in low learning accuracy and a poor classification effect. Currently, there are three main sources of white blood cell image data: (1) own dataset [19]; (2) BCCD original dataset [23–25]; (3) the white blood cell image is generated by the DC-GAN (deep convolutional generative adversarial network) algorithm, the BCCD original data are rotated and cropped, and the two are mixed into a dataset [25]. The own dataset is relatively small, and it is not easy for nonmedical personnel to obtain real white blood cell images; the BCCD original dataset is also relatively small, with only 346 images; since the dataset generated by the DC-GAN algorithm is not real white blood cell imaging, it is still necessary to manually check whether the generated image is close to the real white blood cell. In order to solve the problem of the small white blood cell dataset, the commonly used method is to rotate the image on the basis of the BCCD original dataset to achieve the purpose of expanding the dataset: the first method is to rotate the image horizontally and vertically [25]. Due to the limited rotation angle, the expansion of the dataset is also limited. The second method is to randomly select an angle to rotate the image in the range of 0–360°. This method will greatly expand the dataset, but the rotated image will have a black area, as shown in Figure 1. These black areas have obvious boundaries, which may be used as image features for classification, thereby affecting the classification effect. In order to eliminate the influence of the black area, some researchers have adopted a clipping method to completely remove the black area and retain only the white blood cell image, as shown in Figure 2. This method requires manual intervention and is inefficient. The third method is to multiply the image by the rotation matrix [20]. This method will cause obvious image deformation, resulting in a large change in the morphological characteristics of white blood cells, which in turn affects the classification accuracy, as shown in Figure 3.

In the experimental phase, the impact of a small dataset also exists. Now scholars generally divide the expanded dataset into a training set and a test set in proportion, that is, the test set to verify the effect of the model is the white blood cell images processed by a certain method, not the original image. For example, using the method of randomly rotating the image to expand the dataset, the images in the test set were also rotated and also contain the black area left after the rotation. The real situation is that the images first obtained by medical institutions are all original images that are not rotated. If you want to achieve the effect in the experiment, you need to randomly rotate the original image, which reduces its efficiency.

This paper proposes a new method for expanding the training set of white blood cell images that can achieve the purpose of expanding the training set without manual intervention while retaining the morphological characteristics of white blood cells. First, rotate the white blood cell image randomly, and then use the Canny edge detection algorithm [26] to extract the edge of the black area in the image. Then, count the pixel values that appear most frequently in the unrotated image. Along the edge of the extracted black area, fill the black area in the rotated image with a random value near the pixel value obtained by the above statistics. Finally, obtain an image with the characteristics of the black area eliminated so as to achieve the purpose of expanding the white blood cell image dataset. Use this dataset to train a machine learning model. This paper is organized as follows: Section 2 presents the techniques and methods followed to achieve the research goals; in Section 3, we present experimental results and discussions; the paper concludes in Section 4 at the end.

## 2. Method

This section describes the method of expanding the white blood cell image dataset. In order to ensure the initial characteristics of white blood cells to the greatest extent, this paper rotates the image around the center point as a whole. In order to eliminate the possible influence of the black area caused by rotation on the classification effect, this paper counts the pixels with the most occurrences in the unrotated image and uses a random value near the pixel to fill the black area. The working flow chart of this method is shown in Figure 4.

### 2.1. Image Rotation

The rotation method in this paper takes the image center point as the axis and rotates by a specific angle. The formula is shown in equation (1), where x0, y0, and 1 represent the abscissa, ordinate, and dimension of the pixel after rotation. x, y, and 1 represent the abscissa, ordinate, and dimension before rotation. W and H represent the width and height of the image. *θ* represents the rotation angle. After image rotation, use bilinear interpolation [27] to enhance image quality. The rotated image is shown in Figure 5, and the image is hereinafter referred to as IMG_Rotated.

(1) $$\begin{array}{c} \left[\begin{array}{ccc} X_{0} & Y_{0} & 1 \end{array}\right]=\left[\begin{array}{ccc} X & Y & 1 \end{array}\right]\left[\begin{array}{ccc} \cos\;\theta & -\sin\;\theta & 0\\ \sin\;\theta & \cos\;\theta & 0\\ -0.5W\;\cos\;\theta -0.5H\;\sin\;\theta +0.5W & 0.5W\;\sin\;\theta -0.5H\;\cos\;\theta +0.5H & 1 \end{array}\right]. \end{array}$$

### 2.2. Edge Extraction

After the image is rotated, an obvious black area will appear. Intuitively, the RGB pixel value of this area is #000000. However, when the RGB pixel value of #000000 is used as the judgment condition to fill the black area, it is difficult to fill the edges of the black area, as shown in Figure 6. This paper uses the Canny algorithm to extract the edge of IMG_Rotated, then fill the black area with the edge as the starting point. The Canny algorithm is divided into the following steps:

(1) *Gaussian filter*: For a pixel located at (x,y), its gray value is f(x,y) and the gray value after Gaussian filtering becomes
  (2) $$\begin{array}{c} g_{\sigma }\left(x,y\right)=\frac{1}{\sqrt{2\pi \sigma^{2}}}e^{\left(-x^{2}+y^{2}/2\sigma^{2}\right)}\cdot f\left(x,y\right). \end{array}$$
(2) Calculate gradient value and gradient direction: Calculate the gradients in the horizontal and vertical directions, respectively, and comprehensively obtain the final gradient value and gradient direction, see (3) and (4), where gx(x,y) and gy(x,y) are the gradients in the horizontal and vertical directions, respectively. The result of (4) is the gradient direction.
  (3) $$\begin{array}{c} G\left(x,y\right)=\sqrt{g_{x}{\left(x,y\right)}^{2}+g_{y}{\left(x,y\right)}^{2}}, \end{array}$$
  (4) $$\begin{array}{c} \theta =\arctan\frac{g_{y}\left(x,y\right)}{g_{x}\left(x,y\right)}. \end{array}$$
(3) Filter nonmaximum values.
(4) Use upper and lower thresholds to detect edges.

It sets two thresholds: maxVal and minVal. The pixels above maxVal are detected as edges, and the pixels below minVal are detected as nonedges. For a pixel in the middle, if it is adjacent to a pixel determined to be an edge, it is determined to be an edge; otherwise, it is a nonedge. The edge extracted using the Canny algorithm is shown in Figure 7.

### 2.3. Pixel Filled

There are a lot of monotonous backgrounds in the white blood cell image; see Figure 8. The box is the background, and the pixel value with the most occurrences in the original image is obtained by statistics. We use this pixel value as the pixel value of the image background and use a random value N near the pixel value as the filled pixel value. After obtaining the edge pixels of the black area, count the values of the pixels around the edge pixels and fill in the horizontal or vertical direction with small pixel values until the edge of the image, as shown in Figure 9. The effect of pixel filling is shown in Figure 10. It can be seen from Figure 10(b) that, using the method in this paper, the edges of the black area are well filled.

## 3. Experiment

### 3.1. Experiment Environment

The experimental environment of this paper is as follows:

- CPU: Inter Core i5-11600 KF
- RAM: 16G
- GPU: NVIDIA GEFORCE 1050Ti
- Operating system: Windows 10 64 bit
- *Python*: 3.9
- TensorFlow: 2.6.0

### 3.2. Dataset

This paper uses three sets of datasets, namely, the BCCD original image dataset, the randomly rotated image dataset, and the image dataset processed by the method in this paper. In order to restore the real application scenario, the BCCD original image dataset is divided into a training set and a test set using 10-fold cross-validation. The randomly rotated image and the image dataset processed by the method in this paper are used as the training set, and the BCCD original image dataset is used as the test set, so as to ensure that the test images used are the original, unprocessed white blood cell images when verifying the effect. The datasets are shown in Table 1, the four different types of white blood cells included in the datasets are shown in Figure 11, and the images included in the three datasets are shown in Figure 12.

### 3.3. Evaluation Indicators

In this paper, four parameters: loss, validation accuracy (VA), precision (P), and recall (R), are used as evaluation indicators. This paper uses the cross-entropy loss function, and the calculation formulas for VA, P, and R are shown in equations (5)–(7).

(5) $$\begin{array}{c} VA=\frac{\text{TruePositive}+\text{TrueNegative}}{\text{TotalSamples}}, \end{array}$$

(6) $$\begin{array}{c} P=\frac{\text{TruePositive}}{\text{TruePositive}+\text{FalsePositive}}, \end{array}$$

(7) $$\begin{array}{c} R=\frac{\text{TruePositive}}{\text{TruePositive}+\text{FalseNegative}}. \end{array}$$

### 3.4. Experimental Results and Discussion

This paper uses three models of ResNet50 [28], MobileNet [29], and ShuffleNet [30] to verify the method. Each model is trained for 100 epochs, the learning rate is 0.005, and (n) is 30. The loss value, VA, P, and (r) verification results of each model are shown in Figures 13–24. All the ordinates in the picture are the values obtained during testing.

It can be seen from Figure 13 and 17 that, after training ResNet50 and MobileNet using the dataset generated by the method proposed in this paper, the loss curve of the test is stable, good convergence can be obtained, and the loss value is the smallest. As can be seen from Figure 21, after the ShuffleNet model is trained on the dataset generated by the method proposed in this paper, although the loss value curve fluctuates more than the loss value curve after training with the BCCD original image dataset, the loss value is the smallest in most cases. As can be seen from Figures 13–16, when ResNet50 is trained using the BCCD original image dataset, the loss value of the test cannot achieve good convergence, and the VA, P, and R values have large fluctuations, so a stable prediction effect cannot be obtained. As can be seen from Figure 17, when the BCCD original image dataset trains the MobileNet, the gradient explosion occurs in the 13th epoch loss function, the loss value rises sharply, and its VA, P, and R values all drop significantly. As can be seen from Figure 21, when the ShuffleNet is trained using the rotated image dataset, at the 73th epoch, the loss function has a gradient explosion, the loss value rises sharply, and its VA, P, and R values all drop significantly. Looking at Figures 13–24, using the dataset generated by the method in this paper to train the three models did not experience a gradient explosion. After training with multiple epochs, the loss value, VA, P, and R values can all reach a relatively stable state and have good robustness. When training the ResNet50 and MobileNet, the loss value is the smallest, and the VA, P, and R values are the largest. When training the ShuffleNet, the loss value is also the smallest most of the time, and the VA, P, and *R* values are the largest.

We use (8) to make a quantitative evaluation of the improvement in loss, VA, P, and R values. Based on the loss value, VA, P, and R values obtained by training the three models on the BCCD original image dataset, calculate the value of each parameter improvement of the 20 epochs after stabilization; this paper uses the 80th epoch to the 100th epoch. *Pan* is the loss value, VA, P, or R at the nth epoch using the rotated image dataset or the dataset generated by the method in this paper; Bn is the loss value, VA, P, or R at the nth epoch using the BCCD original dataset; the total training times of epochs and the results are shown in Table 2–4.

(8) $$\begin{array}{c} I=\frac{\sum_{n=i}^{i+19}\left(\left(Pa_{n}-B_{n}\right)/B_{n}\right)}{20}. \end{array}$$

It can be seen from Table 2–4 that when the rotated image dataset is compared with the original BCCD dataset, the VA, P, and R values are significantly improved, except that the loss value in the ShuffleNet is not improved. Using the dataset generated by the method in this paper to train the three models, the loss value, VA, P, and R values are further improved compared with the rotated image dataset.

## 4. Conclusion

White blood cell image classification based on machine learning has important clinical significance, but for nonmedical practitioners, it is difficult to obtain white blood cell image datasets for training and learning, and the size of the dataset affects the training and validation of the model. This paper proposes a white blood cell dataset expansion method, which uses the black area edges that appear after image rotation and the original image pixels to count and fill the black area, so as to reduce the possibility of the black area generated by rotation as a feature affecting the classification effect. Experiments show that the dataset obtained by using the method in this paper is used for ResNet, MobileNet, and ShuffleNet training, and the model obtained by training has better robustness and the prediction accuracy is significantly improved.

The main idea of the method in this paper is to use white blood cell images with a large number of monotonous backgrounds; image rotation will produce black areas, and the obvious edges between this area and the original image; fill the black area with pixels from the edge as the starting point, and then study images with the same characteristics in other fields to study the possibility of applying this algorithm in other fields.

## Figures and Tables

**Figure 1:** Rotated image.

**Figure 2:** Cropped image.

**Figure 3:** Image rotated by rotation matrix.

**Figure 4:** Working flow chart.

**Figure 5:** Rotated image.

**Figure 6:** Fill black area directly. (a) The image obtained by directly filling the area with the RGB pixel value of #000000. (b) The image obtained by directly filling areas with pixel values below 30.

**Figure 7:** (a) The image of rotated white blood cells. (b) The image after extracting black area edges using Canny.

**Figure 8:** Original image of white blood cells.

**Figure 9:** Fill black area (the arrow is the fill direction, it is also possible to fill in the vertical direction).

**Figure 10:** Filled white blood cell image.

**Figure 11:** Images from three datasets. (a) The BCCD original image. (b) The randomly rotated image. (c) The image processed by the method in this paper.

**Figure 12:** Four different types of white blood cells. (a) Eosinophil. (b) Monocyte. (c) Lymphocyte. (d) Neutrophil.

**Figure 13:** ResNet50 model loss value curve.

**Figure 14:** ResNet50 model VA value curve.

**Figure 15:** ResNet50 model *P* value curve.

**Figure 16:** ResNet50 model *R* value curve.

**Figure 17:** MobileNet model loss value curve.

**Figure 18:** MobileNet model VA value curve.

**Figure 19:** MobileNet model *P* value curve.

**Figure 20:** MobileNet model *R* value curve.

**Figure 21:** ShuffleNet model loss value curve.

**Figure 22:** ShuffleNet model VA value curve.

**Figure 23:** ShuffleNet model *P* value curve.

**Figure 24:** ShuffleNet model *R* value curve.

**Table 1:** Datasets.

		BCCD original image dataset	Randomly rotated image dataset	Image dataset processed by the algorithm in this paper
Training set	Eosinophil	79	2497	2497
	Lymphocyte	30	2483	2483
	Monocyte	18	2478	2478
	Neutrophil	185	2499	2499
Total		312	346	346

Test set	Eosinophil	8	87	87
	Lymphocyte	3	33	33
	Monocyte	2	20	20
	Neutrophil	21	206	206
Total		34	346 (all from the BCCD original dataset)	346 (all from the BCCD original dataset)

**Table 2:** The effect of ResNet improvement.

	Using rotated image dataset	Using the dataset generated by the method in this paper
Loss	−61.4%	−74.07%
VA	181.84%	194.69%
P	186.49%	198.89%
R	206.01%	221.14%

**Table 3:** The effect of MobileNet improvement.

	Using rotated image dataset	Using the dataset generated by the method in this paper
Loss	−29.96%	−34%
VA	126.89%	143.29%
P	127.93%	145.06%
R	124.84%	141.95%

**Table 4:** The effect of ShuffleNet improvement.

	Using rotated image dataset (%)	Using the dataset generated by the method in this paper (%)
Loss	54.77	35.31
VA	74.24	93.98
P	70.64	91.15
R	73.49	92.88

## Data Availability

The data used to support the findings of this study are included within the article.
